# Comparison of the Application Value for Diagnosis of Chronic Kidney Disease between Color Doppler Flow Quantification Technique and Computed Tomography

**DOI:** 10.1155/2022/6485273

**Published:** 2022-07-08

**Authors:** Yusen Zhao, Renzhong Zhang, Yaoyi Wang, Yuanbo Xu, Xiangming Wang

**Affiliations:** ^1^Department of Medical Imaging, The First Affiliated Hospital of Hebei North University, Zhangjiakou 075000, Hebei, China; ^2^Departmrnt of Nephrology, Zibo Central Hospital, Zibo 255000, Shandong, China; ^3^Center of Returning Visit, The First Affiliated Hospital of Hebei North University, Zhangjiakou 075000, Hebei, China; ^4^Department of CT Magnetic Resonance, The Fourth Hospital of Hebei Medical University, Shijiazhuang 050000, Hebei, China

## Abstract

**Objective:**

The aim of this study is to compare the application value for diagnosis of chronic kidney disease (CKD) between the color Doppler flow quantification (CDFQ) technique and computed tomography (CT).

**Methods:**

The clinical data of 88 hospitalized patients treated in the Renal Medicine of our hospital and diagnosed with CKD after pathological examination from June 2020 to June 2021 were selected for the retrospective analysis, and 32 individuals with normal physical examination results in the same period were selected as the control group. All study subjects received CDFQ and 640-slice volume CT examination, and by plotting the ROC curves, the clinical value of different diagnostic modalities was analyzed.

**Results:**

The 3D renal volumes between the stage 1 group and control group were significantly different (*P* < 0.05); the 3D renal volumes between the stage 2 group and control group and between the stage 2 group and stage 1 group were significantly different (*P* < 0.05); in the comparison between the stage 3 group versus control group/stage 2 group, the RI values, 3D renal volumes, and cortical thicknesses were significantly different (*P* < 0.05); in the comparison between the stage 4 group versus control group/stage 1 group, the RI values, 3D renal volumes, and cortical thicknesses were significantly different, and between the stage 4 group and stage 2 group, the RI values and cortical thicknesses were significantly different (*P* < 0.05); in the comparison between the stage 5 group versus control group/stage 1 group/stage 2 group/stage 3 group, the RI values, 3D renal volumes, and cortical thicknesses were significantly different, and between the stage 5 group and stage 4 group, the RI values and 3D renal volumes were significantly different (*P* < 0.05); among various groups, the measurement indicators of 640-slice volume CT scan were significantly different (*P* < 0.05); and in terms of disease classification, the AUC value, positive predictive value, negative predictive value, sensitivity, and specificity of 640-slice volume CT were higher than those of CDFQ diagnosis.

**Conclusion:**

640-slice volume CT has a higher efficacy in diagnosing CKD and can provide a reliable basis for the selection of treatment schemes for CKD patients.

## 1. Introduction

The kidney is one of the vital organs in the human body as well as the target organ of many diseases [1]. Chronic kidney disease (CKD) is a common clinical condition with the common clinical manifestations such as nausea, vomiting, loss of appetite, and dysuria and has been widely concerned because of its high incidence, long disease duration, and poor clinical outcomes. CKD has complicated pathogenic factors and irreversible pathological development; renal needle biopsy is currently the common way to diagnose CKD, but it is one of the invasive examinations [2, 3], with an odd choice of puncture point and a certain risk of infection and bleeding, and repeated operation is not suitable, so there are limitations in clinical diagnosis. Therefore, it is of great significance to seek efficient clinical diagnostic modalities [4]. Recently, with the development of medical imaging technology, the color Doppler flow quantification (CDFQ) technique has been used in clinic as a diagnostic modality that is noninvasive, safe, convenient, and effective for the quantitative evaluation of renal cortical hemoperfusion [5], which can be used for splanchnic blood flow perfusion assessment and has the clinical characteristics such as easy operation, low price, and reusability [6]. In recent years, many scholars at home and abroad have done many explorations on computerized tomography (CT) in the evaluation of renal function and obtained a more recognized clinical value in the diagnosis of diseases including small kidney stones [7]. 640-slice volume CT is equipped with an ultrawide detector, and its ultrahigh speed volume scanning technology can complete a full circle scan in 0.35s, thus avoiding scanning errors caused by patient position shifting during helical scanning and unnecessary radiation, which has a certain clinical significance in the evaluation of renal function [8]. CKD can seriously affect the renal function of patients. This study provided a reliable basis for valid diagnosis of CKD and the development of treatment options to improve the quality of life of patients, offering a theoretical support for future in-depth studies. In this study, the efficacy of diagnosing CKD by CDFQ and 640-slice volume CT was compared, providing a new direction for the diagnosis of CKD.

## 2. Materials and Methods

### 2.1. General Data

The clinical data of 88 hospitalized patients treated in the Renal Medicine of our hospital and diagnosed with CKD after pathological examination from June 2020 to June 2021 were selected for the retrospective analysis, and 32 individuals with normal physical examination results in the same period were selected as the control group. The study was approved by the hospital ethics committee and met the World Medical Association Declaration of Helsinki [9]. In the CKD group, there were 54 males and 34 females, the patients' age range was 32–65 years, and the mean age was (49.40 ± 9.93) years. The staging was conducted according to the clinical standard staging method as follows. (1) Stage 1: normal glomerular filtration rate (GFR), ≥90 ml·min^−1^· (1.73 m^2^)^−1^; (2) stage 2: slightly abnormal GFR, 60–89 ml·min^−1^ (1.73 m^2^)^−1^; (3) stage 3: moderately abnormal GFR, 30–59 ml·min^−1^· (1.73 m^2^)^−1^; (4) stage 4: severely abnormal GFR, 15–29 ml·min^−1^·(1.73 m^2^)^−1^; and (5) stage 5: renal failure could be determined initially. Among the CKD patients, 23 cases were at stage 1, 20 cases were at stage 2, 16 cases were at stage 3, 13 cases were at stage 4, and 16 cases were at stage 5. A total of 32 healthy individuals with normal results of physical examinations (routine urine test and renal function test) in the same period were selected as the control group, including 18 males and 14 females, their age range was 33–67 years, and their mean age was (49.59 ± 10.03) years. Inclusion criteria were as follows: no contraindications of CDFQ and CT examination; exclusion criteria were as follows: (1) those with abnormal renal structure (medullary sponge kidney, polycystic kidney); (2) those with stenosis of renal artery; and (3) those who had obesity, hydronephrosis, and with poor compliance.

### 2.2. Diagnostic Modalities

CDFQ diagnosis. The CTS-5500 ultrasonic diagnostic apparatus (manufacturer: Hubei Renxu Medical Instrument Co., Ltd.) was used with the frequency set as 3–5 MHz. The patients were told to lie on the side to connect with the electrocardiogram machine, the routine ultrasound was performed to show the maximum section of kidney and fully show the renal hilum, and the distance from the superior border of renal to body surface was kept as 5 cm. The patients were told to hold their breath, the color Doppler mode was initiated, the sampling frame contained the entire kidney to dynamically observe the intrarenal color flow signal distribution, intensity, and blood flow stream continuity, and at the same time, the color blood flow dynamic images of 3 cardiac cycles were dynamically stored for subsequent analysis.

640-slice volume CT examination. The scanning equipment was Toshiba Aquilion One 640-slice volume CT machine. Before examination, the patients were told to fast and drink 1,000 ml of water, hold the urine until bladder filling, and lie on their back on the examination bed to do the respiratory training. The patients kept the supine position, foot first was selected, and volume scanning mode and helical scanning mode were selected to scan the area from the upper pole of both kidneys (including bilateral adrenal gland) to the anterior superior iliac spine.

### 2.3. Image Analysis

CDFQ. The region of interest (ROI) was analyzed with analysis software Q-LAB10, a cardiac cycle was selected, the ROI sampling frame contained the entire kidney, the peripheral tissue entering into the ROI was avoided, and the 3D renal volume, cortical thickness, and interlobar artery resistance index (RI) were automatically generated by the software.

640-slice volume CT. After the end of examination, image measurement was performed in the GE ADW46 workstation, and the measurement indexes included CT values in the cortical phase, medullary phase, and lag phase.

### 2.4. Statistical Methods

The statistic software SPSS26.0 was used, the enumeration data were examined by *χ*^2^ test and expressed by (*n*(%)), the measurement data were examined by *t*-test and expressed by Mean ± SD, and differences were considered statistically significant at *P* < 0.05.

## 3. Results

### 3.1. Comparison of CDFQ Observation Indexes among Various Groups

In the comparison between the stage 1 group versus control group, the 3D renal volumes were significantly different (*P* < 0.05); in the comparison between the stage 2 group versus control group/stage 1 group, the 3D renal volumes were significantly different (*P* < 0.05); in the comparison between the stage 3 group versus control group/stage 2 group, the RI values, 3D renal volumes, and cortical thicknesses were significantly different (*P* < 0.05); in the comparison between the stage 4 group versus control group/stage 1 group, the RI values, 3D renal volumes, and cortical thicknesses were significantly different, and in the comparison between the stage 4 group and stage 2 group, the RI values and cortical thicknesses were significantly different (*P* < 0.05); in the comparison between the stage 5 group versus control group/stage 1 group/stage 2 group/stage 3 group, the RI values, 3D renal volumes, and cortical thicknesses were significantly different, and in the comparison between the stage 5 group versus stage 4 group, the RI values and 3D renal volumes were significantly different (*P* < 0.05). See Table 1.

### 3.2. Comparison of Various Measurement Indexes of 640-Slice Volume CT Scan among Various Groups

The study results found that the measurement indexes of 640-slice volume CT scan among various groups were significantly different (*P* < 0.05). See Table 2.

### 3.3. Comparison of the Diagnostic Value for Different Types of CDK between the Two Diagnosis Modalities

In different disease types, the AUC value, positive predictive value, negative predictive value, sensitivity, and specificity of 640-slice volume CT were higher than those of CDFQ diagnosis. See Table 3 and Figure 1.

## 4. Discussion

CKD is a class of common diseases with continuous progression and common clinical manifestations including dysuria, loss of appetite, and nausea, and data from multicenter studies have shown [10–12] that the prevalence of CKD in the population is up to 10.8%, and most patients with stage 1–3 CKD are asymptomatic and can progress to end-stage renal disease without any signs. The renal pathological changes in CKD are glomerular fibrosis and sclerosis, glomerular atrophy and degeneration, interstitial fibrosis, inflammatory cell infiltration, thickening of the tubular wall of renal arterioles, and hyaline degeneration, which lead to increased renal artery resistance, decreased renal blood flow perfusion, thinner renal cortex, reduced GFR, and then renal dysfunction. With progression of the disease, all levels of renal blood vessels are involved, so intrarenal blood flow perfusion and disease progression are closely related. Therefore, early diagnosis and treatment are particularly critical to improve the prognosis of CKD [13–15].

Current imaging modalities for the diagnosis of CKD mainly include radionuclide scanning, MRI, CT, and ultrasonic contrast [16]. Radionuclide scanning can assess the patients' renal blood flow perfusion, GFR of the total and split kidneys, upper urinary tract patency, and other comprehensive information, but this diagnostic technique is radiological and cannot be manipulated repeatedly [17]. Some scholars believe [18] that the CDFQ diagnostic technique can be used for splanchnic blood perfusion assessment, which is a new diagnostic method formed based on the conventional two-dimensional ultrasound and color Doppler technology and can quantitatively assess renal blood perfusion by using professional software analysis, which is easy, quick, inexpensive, and can be reused multiple times [19, 20]. However, 640-slice volume CT can precisely localize the renal lesions in patients and has diagnostic advantages such as high resolution and multislice imaging, as well as rapid detection of renal tumor lymph node metastasis and signs such as infiltration and deep venous tumor thrombus, but the inability of dynamic observation as well as radiopacity make its clinical application limited [21]. The diagnostic value of virtual touch quantification (VTQ) in CKD has been affirmed by the latest study [22], but it only analyzed the rate of positive disease diagnosis and lacked research on various imaging parameters. In this study, the clinical data of 88 patients diagnosed with CKD after pathological examination were selected for the retrospective analysis and 32 individuals with normal physical examination results in the same period were selected as the control group, and by performing CDFQ and CT diagnosis to the study subjects, the diagnostic efficacy of different diagnosis modalities was analyzed, providing valuable reference for the early diagnosis of CKD in clinic. After analyzing the data in Table 1, it could be concluded that the three-dimensional renal volumes between the control group and the patients at all stages were significantly different (*P* < 0.05), indicating that when a lesion or inflammatory reaction occurs in the kidney, it would cause a significant change in renal volume, which also provides a direction for subsequent diagnosis. Some scholars [23] only explored the positive predictive value and accuracy of CT in the diagnosis of CKD in their studies, while the related diagnostic data obtained in this study were more comprehensive, making it one of the strengths of this study. The study results confirmed that in the clinical diagnosis of CKD at different stages, the AUC value, sensitivity, specificity, and other indicators of 640-slice volume CT were higher than those of CDFQ diagnosis, and the reason might be that 640-slice volume CT scan is an imaging diagnostic technique that integrates anatomy and function, which can accomplish the “one-stop” evaluation of organs, greatly improve the temporal and spatial resolution, also ensure the image definition, and without the need for increasing the amount of additional radiation dose and contrast agent, complete comprehensive evaluation of renal function, presenting its value for the diagnosis and treatment of CKD; whereas, the results of CDFQ are greatly related to the skill of the examining physician, which combined with its image definition and resolution lower than 640-slice volume CT, results in limitations in diagnosis [24, 25]. The contributions of the study were as follows: it aimed to provide a well-established and efficient diagnostic scheme for patients and the basis for developing a precise clinical treatment plan by implementing CDFQ versus CT diagnosis for CKD patients and comparing imaging indexes of patients at all stages, which is a great advance and development of clinical imaging diagnosis, has a broad guidance in modern diagnosis of renal diseases, and is undoubtedly a future direction of medicine.

In conclusion, 640-slice volume CT can effectively improve the accuracy of diagnosing CKD, with clinical diagnostic efficacy better than that of CDFQ diagnosis, so it is expected to be the effective method for early diagnosis of CKD, dynamic monitoring of disease progression, and evaluation of clinical efficacy and prognosis. However, the study also had some shortcomings, for example, the sample size included was smaller, which might cause bias in the results, and the factors such as age and complications on results were not considered. Hence, the trial design should be further improved and the sample size should be expanded in the future studies to provide more accurate clinical basis for the diagnosis of CKD. Although modern medical diagnosis technology is continuously progressing, there are still many dilemmas in the diagnosis of CKD. Therefore, as medical workers, we still need to make continuous efforts to explore more efficient diagnosis technology, optimize the current diagnosis mode, and provide reliable data support for the diagnosis of CKD. It is believed that with the constant development of technologies, the imaging examination will have a more profound impact on the diagnosis and treatment of CKD, and more CKD patients will benefit from it in the future.

## Figures and Tables

**Figure 1:** ROC curves of different types of CDK by the two diagnostic modalities. A-E show the ROC curves of stages 1, 2, 3, 4, and 5 of CDK by the two imaging modalities.

**Table 1:** Comparison of CDFQ observation indexes among various groups (Mean ± SD).

Group	*n*	Cortical thickness (mm)	3D renal volume (ml)	RI
Control	32	0.95 ± 0.05	146.34 ± 14.32	0.61 ± 0.05
Stage 1	23	0.98 ± 0.06	166.09 ± 21.77^a^	0.64 ± 0.04
Stage 2	20	0.96 ± 0.04	134.30 ± 13.70^b^	0.63 ± 0.05
Stage 3	16	0.84 ± 0.05^abc^	127.69 ± 15.26^ab^	0.66 ± 0.03^abc^
Stage 4	13	0.78 ± 0.05^abc^	119.23 ± 12.83^ab^	0.69 ± 0.04^abc^
Stage 5	16	0.62 ± 0.04^abcde^	111.44 ± 11.67^abcde^	0.71 ± 0.05^abcde^

a indicates *P* < 0.05 versus control group; b indicates *P* < 0.05 versus stage 1 group; c indicates *P* < 0.05versus stage 2 group; d indicates *P* < 0.05versus stage 3 group, and e indicates *P* < 0.05 versus stage 4 group.

**Table 2:** Comparison of various measurement indexes of 640-slice volume CT scan among various groups (Mean ± SD).

Group	*n*	CT values in the lag phase (HU)	CT values in the cortical phase (HU)	CT values in the medullary phase (HU)
Control	32	145.13 ± 5.05	206.38 ± 8.63	181.47 ± 6.01
Stage 1	23	135.13 ± 4.99^a^	179.57 ± 3.55^a^	172.09 ± 5.99^a^
Stage 2	20	127.90 ± 5.17^ab^	158.05 ± 3.89^ab^	161.25 ± 6.60^ab^
Stage 3	16	120.44 ± 4.94^abc^	140.56 ± 7.48^abc^	152.69 ± 5.92^abc^
Stage 4	13	114.31 ± 2.63^abcd^	131.54 ± 4.27^abcd^	137.23 ± 4.88^abcd^
Stage 5	16	97.44 ± 5.91^abcde^	117.38 ± 5.54^abcde^	122.94 ± 5.79^abcde^

a indicates *P* < 0.05 versus control group; b indicates *P* < 0.05versus stage 1 group; c indicates *P* < 0.05 versus stage 2 group; d indicates *P* < 0.05versus stage 3 group, and e indicates *P* < 0.05versus stage 4 group.

**Table 3:** Comparison of the diagnostic value for different types of CDK between the two diagnosis modalities.

Group	AUC value		Positive predictive value		Negative predictive value		Sensitivity		Specificity	
	640-slice volume CT	CDFQ	640-slice volume CT	CDFQ	640-slice volume CT	CDFQ	640-slice volume CT	CDFQ	640-slice volume CT	CDFQ
Stage 1	0.835	0.636	82.61%	52.17%	84.38%	75.00%	79.17%	60.00%	87.10%	68.57%
Stage 2	0.822	0.675	80.00%	60.00%	84.38%	75.00%	76.19%	60.00%	87.10%	75.00%
Stage 3	0.875	0.799	87.50%	75.00%	87.50%	84.38%	77.78%	70.59%	93.33%	87.10%
Stage 4	0.822	0.791	76.92%	76.92%	87.50%	81.25%	71.43%	62.50%	90.32%	89.66%
Stage 5	0.813	0.750	75.00%	68.75%	87.50%	81.25%	75.00%	64.71%	87.50%	83.87%

## Data Availability

The data used to support the findings of this study are available on reasonable request from the corresponding author.
